# Effect of Hand Intensive Training on Upper Limb Function of Stroke Patients with Hemiplegia

**DOI:** 10.1155/2022/6844680

**Published:** 2022-03-25

**Authors:** Xiaoxia Gou, Xian Zhang, Xiaxia Zheng, Yaozhong Zhang, Hongxiang Ma

**Affiliations:** ^1^Department of Neurology, Lanzhou University Second Hospital, Lanzhou, 730000 Gansu, China; ^2^Department of Rehabilitation Medicine, Lanzhou University Second Hospital, Lanzhou, 730000 Gansu, China

## Abstract

**Objective:**

To analyze the effect of hand intensive training on upper limb function of stroke patients with hemiplegia,

**Methods:**

110 stroke patients were randomly divided into two groups: the reference group and the observation group. 55 patients in the reference group were treated with routine rehabilitation treatment, including routine joint activity training, bed training, exercise therapy, and ADL ability training; 55 cases in the observation group received intensive hand training on the basis of routine rehabilitation treatment, including inducing the patient's five finger extension, forcibly pulling the fingers and wrist joints, and suddenly opening his fist after clenching his fist.

**Results:**

The treatment period of the two groups was 5 weeks. In the comparison results of Fugl-Meyer (FMA), the exercise effect of the observation group with increased hand intensive training was significantly better than that of the control group with stroke hemiplegia treated with conventional methods. The difference was statistically significant, *t* < 10.000, *P* < 0.05; In the comparative analysis of upper limb function test (UEFT), the effect of the observation group was significantly higher than that of the reference group treated with routine rehabilitation nursing (all *P* < 0.05); In the comprehensive comparison of exercise ability results, the observation group was higher than the reference group in the flexibility, fineness, and fineness of activity behavior after treatment.

**Conclusion:**

Strengthening hand intensive training can further improve the upper limb motor function of stroke patients with hemiplegia, reduce the severity of hemiplegia, and improve the recovery effect of stroke patients. It is worthy of clinical promotion and application.

## 1. Introduction

In China, the incidence rate of stroke is increasing, and it has become one of the important causes of limb dysfunction and high disability rate in our country. Therefore, stroke can lead to disability even if patients recover. Moreover, the age of onset of the disease is also younger and increasing year by year, which has seriously affected people's physical and mental health, but there is a lack of very effective treatment at present. Therefore, it is considered that early prevention is a very good measure to eliminate the incidence of stroke from the source. This study analyzes and discusses the influence of hand intensive exercise on the function of left and right limbs of upper body of stroke hemiplegic patients (NZZPTHZ) and compares the clinical technical research on the influence of relevant methods of hand limb intensive training on the function of upper body limbs of stroke hemiplegic patients (NZZPTHZ).

“Stroke” is the blockage of blood vessels in the brain. It is an acute cerebrovascular disease. It is a general term and common name for acute cerebrovascular diseases. It is also known as cerebrovascular accident. Clinically, it mainly includes cerebral infarction, thrombosis, intracerebral hemorrhage, and other diseases. The incidence rate of stroke patients has been increasing year by year in recent years. Most stroke patients can maintain vital signs or recovery after rescue treatment, but even after recovery, there are generally different degrees of dysfunction, especially hemiplegia (hemiplegia). Ying et al. [1] pointed out that stroke is the most serious brain disease problem in stroke patients with hemiplegia and is also the most important cause of disability and death in adults. According to the survey, the incidence rate of stroke in China is 403.08/10 million in recent years, of which 80% of stroke patients will cause limb dysfunction after the onset. The injury of upper limb function is more serious [1]. Feng analyzed the clinical impact of rehabilitation training on NZZPTHZ hand and joint function and daily life self-care ability, saying that 75% of stroke patients will be accompanied by functional disorders such as hand dysfunction and upper limb dysfunction, which has brought serious inconvenience to patients' daily life and seriously caused the physical and mental burden of patients and their families [2]. Yu et al. analyzed the effect of rehabilitation of upper left and right limbs on the rehabilitation of upper limb motor ability of NZZPTHZ, they believe that the rehabilitation training system of the upper limb can effectively improve the motor function of the upper left and right limbs of NZZPTHZ and improve the clinical rehabilitation effect [3]. Zhiying et al. also believe that through the evaluation results of relevant indicators, enhancing the motor ability of upper left and right limb functions has good social recognition and can be used for the clinical application evaluation of NZZPTHZ upper limb function [4]. The deficiency of the above literature review is the lack of a targeted intensive training method to study the effect of upper limb function in stroke patients with hemiplegia.

The main research direction of this study is to analyze the impact of hand intensive training on upper limb function of stroke patients with hemiplegia and comprehensively compare the relevant clinical medical test data, market research, and posttraining recovery effect, so as to explore the application advantages of hand intensive training method in upper limb function of stroke patients with hemiplegia.

## 2. Data and Methods

### 2.1. Clinical Data

110 stroke hemiplegic patients hospitalized in the Department of Neurology and Brain Surgery of an Affiliated Hospital in Jiangsu from January 2021 to June 2021 were selected. There were 60 males and 50 females, aged from 33 to 67 years, with an average of 41.37 ± 2.51 years. The course of disease ranged from 7 to 34 days, with an average of 22.46 ± 2.37 days. All 110 patients had no audio-visual and understanding impairment and had varying degrees of hemiplegia. Inclusion criteria include patients with primary stroke diagnosed by brain CT or MRI and relevant clinical diagnostic criteria; Exclusion criteria include patients with worsening condition; new cerebral infarction or bleeding; comprehensive dysfunction symptoms of important organs such as the heart, liver, and lung; visual space disorder; and unable to tolerate daily intensive training [8]. All patients signed informed consent and the experiment was approved by the ethics committee of the hospital. NZZPTHZ and the analysis results of admission diagnosis are shown in Figure 1.

In Figure 1, the incidence of stroke sequelae caused by cerebral nerve infarction, cerebral vascular embolism, and lacunar infarction is higher than that of stroke patients. Cerebral nerve infarction, cerebral vascular embolism, and lacunar infarction all belong to ischemic stroke. The main reason is the edema of nerve tissue caused by ischemia, and the patient has the symptoms of ischemia and hypoxia. Its incidence is higher than that of intracerebral hemorrhage in patients with hemorrhagic stroke, such as subarachnoid hemorrhage.

### 2.2. Grouping and Methods

110 cases NZZPTHZ were randomly divided into two groups: the reference group and the observation group. There were 55 patients in the reference group, 34 males and 21 females, with an average age of 39 ± 4.6 years; 55 cases in the observation group, 35 males and 20 females; The average age was 44 ± 3.8 years. The reference group received routine rehabilitation treatment, including routine joint activity training, bed training, exercise therapy, ADL ability training, sit to stand training, twice a day, 40 minutes each time. On the basis of routine rehabilitation treatment, the observation group increased hand intensive training methods, including inducing the patient's five finger extension, forcibly pulling fingers and wrist joints, and suddenly opening after clenching his fist and taking the initiative to strengthen exercise, such as taking the cup on the table with the hemiplegic hand, taking beans or food with chopsticks, once a day, about 20 minutes each time, and the treatment cycle is 5 weeks [9]. In order to analyze the pathological causes of stroke patients in more detail, the clinical history data of the above stroke patients are analyzed, as shown in Table 1.

Table 1 shows that among stroke patients, the proportion of male patients is higher than that of female patients, the prevalence of smoking history is also higher, and the age of patients tends to be younger. The prevalence of hypertension, diabetes, hyperlipidemia, and other common diseases is also significantly higher. Therefore, it is of great significance to strengthen early rehabilitation nursing for stroke patients with hemiplegia.

### 2.3. Statistical Methods

The process of analyzing the effect of finger and joint intensive training on the motor function of upper limb NZZPTHZ involves relevant data and indexes. It is necessary to use statistical bivariate *t*-test to compare the differences of relevant data and indicators. Among them, value is *t* value. When *t* < 10.000, it is considered that there is a statistical difference. The smaller *t* value, the greater the statistical difference; Log value is *P* value. When *P* < 0.05, it is considered to have statistical reliability, and when *P* < 0.01, it is considered to have statistical significance; The calculation formula of *t* value is as follows (1):

(1) $$\begin{array}{c} t_{\text{Value}}=\frac{\sum_{i=1}^{n}\left(x_{i}-{\tilde{x}}_{i}\right)}{\sum_{i=1}^{n}\left(x_{i}-\bar{x}\right)}, \end{array}$$

where *t*_Value_ is the output results for *t* value; ${\tilde{x}}_{i}$is the *x*_*i*_ control value after regression; and $\bar{x}$ is the arithmetic mean of statistical sequence *x*,

## 3. Results

### 3.1. Comparison of Fugl-Meyer Evaluation of Motor Function between the Two Groups

The two groups NZZPTHZ used Fugl-Meyer (FMA) for comparative analysis in motor rehabilitation treatment. FMA is a method to evaluate sensorimotor dysfunction in stroke patients. After many tests, it has been widely used in the clinical evaluation of physical motor function [10]. For the two groups NZZPTHZ, the evaluation and comparison of motor function of the upper left and right limbs before and after nursing treatment are shown in Table 2.

Table 2 shows that in the comparison of upper limb motor function of stroke patients, the exercise effect of the observation group treated with intensive training of the fingers and joints is significantly better than that of the reference group treated with conventional methods NZZPTHZ. There was significant difference between the two groups, *t* < 10.000, *P* < 0.05.

In order to better reflect the Fugl-Meyer evaluation and comparison results of motor function between the two groups, the experimental data were visualized, as shown in Figure 2.

In Figure 2, the motor function comparison results of the observation group after treatment are significantly better than those of the reference group, which can improve the influence of upper limb function of hemiplegic patients and has clinical application value.

### 3.2. Comparison of Upper Limb Function Test (UEFT) Evaluation between the Two Groups

The two groups of stroke patients were compared and analyzed by upper left and right limb function test UEFT after 5 weeks of rehabilitation treatment. The evaluation of UEFT scale is not only a simple and practical method for upper limb function evaluation but also a comprehensive evaluation of individual subjective factors of stroke patients [11, 12]. The evaluation and comparison results of upper left and right limb function test UEFT between the two groups are shown in Table 3.

In Table 3, it is obvious that the upper limb function test UEFT evaluation of stroke hemiplegic patients after intensive hand training is higher than that of the reference group treated with routine rehabilitation nursing, and the effect is significant (all *P* < 0.05), which is statistically significant.

According to the results of upper limb function test UEFT evaluation and comparison data of the two groups, the relevant experimental data are visualized, as shown in Figure 3.

Figure 3 shows that the effect of the observation group in the evaluation and comparison of upper left and right limb function test UEFT is better than that of the reference group, and the effect is significant. It shows that strengthening the intensive training of the hands and joints can significantly improve the motor function of the upper body of stroke patients and reduce the severity of hemiplegia.

### 3.3. Comparison of Comprehensive Exercise Performance between the Two Groups

In order to compare the upper limb motor function of the two groups of stroke patients in more detail, the flexibility, fineness, and coordination of hemiplegic patients were compared after treatment. The comprehensive comparison results of the two groups are shown in Table 4.

The comparison result data of the two groups in Table 4 are visualized to obtain a more intuitive comprehensive comparison result of motor ability, as shown in Figure 4.

Table 4 and Figure 4 show that in the comprehensive comparison of motor ability results between the two groups of stroke patients, the flexibility, fineness, and fineness of activity behavior in the observation group are higher than those in the reference group after treatment. It shows that strengthening the intensive training of the hands and related joints can improve the recovery effect of NZZPTHZ.

## 4. Discussion

Through the analysis of the effect of hand intensive training on the upper limb function of (NZZPTHZ), this study conducted Fugl-Meyer (FMA), upper limb function test (UEFT), and the flexibility, fineness of using chopsticks, placing building blocks, and picking beans in the exercise rehabilitation treatment for the two groups of stroke patients with the same course of rehabilitation treatment but different methods. After the comparison of coordination and other indicators, the data differences between the two groups are obtained, which shows that the recovery of motor function of NZZPTHZ is better than that of patients with routine rehabilitation treatment. Jia et al. studied the progress of compulsory exercise therapy in the rehabilitation treatment of stroke hemiplegia and believed that in the application of compulsory exercise therapy in functional training and rehabilitation exercise of hemiplegic patients, based on the combination theory of brain plasticity and brain function, intensive training can improve the daily activity ability and motor function of stroke patients [5, 13]. Ankang said in the study of predicting upper limb motor function after stroke that abnormal proprioception of the affected upper limb can reflect the prognostic factors of upper limb motor function after stroke and improve the recovery of upper limb motor function after stroke [6, 14]. Xiaoxia et al. in the impact of mandatory exercise therapy on the recovery of upper limb motor function in patients with poststroke hemiplegia, they believe that mandatory exercise therapy can assist patients with poststroke hemiplegia and have a positive impact on the recovery of upper limb function and the improvement of daily living ability, and the clinical effect is significant [7, 15]. The above related studies show that the training method of upper limb motor function can contribute to the rehabilitation effect of stroke patients, but due to the complexity of human hand motor function system, the recovery of hand function is also slow, which affects the rehabilitation effect of patients.

This study adds the hand intensive training method to the traditional rehabilitation treatment of stroke patients with hemiplegia, which can not only exercise the hand function of patients, that is, the drafting activities of the finger joints and other parts, but also effectively stimulate the motor nervous system of patients, increase the mobility of skeletal muscles, and improve the motor ability of the upper limbs. After intensive hand training, the upper limb motor function of patients is significantly improved compared with the previous one, which reduces the patient's condition, plays an important clinical role in early recovery, is beneficial to the patient's mental health, and improves the patient's quality of life.

## 5. Summary

The purpose of this study is to study the effect of hand intensive training on the upper limb function of stroke patients with hemiplegia. The data from this study show that hand intensive training is added on the basis of traditional rehabilitation treatment, which has a leading effect on the upper limb function of stroke patients with hemiplegia, creating conditions for early rehabilitation care and repair, so that the damaged neuromotor system can restore the motor function of the limbs under the stimulation of intensive training [16]. This is also the extended application of comprehensive rehabilitation treatment for stroke patients with hemiplegia, which can prevent complications, promote the recovery of motor function, take care of themselves, and improve the quality of life. In conclusion, strengthening hand intensive training has the clinical significance of early rehabilitation nursing for stroke patients with hemiplegia.

## Figures and Tables

**Figure 1:** Analysis results of admission diagnosis and etiology of stroke patients.

**Figure 2:** Visual comparison of FMA function results of the upper limbs between the two groups before and after treatment.

**Figure 3:** Visualization of evaluation and comparison results of upper limb function test UEFT between the two groups.

**Figure 4:** Visual diagram of comprehensive comparison of exercise ability results between the two groups.

**Table 1:** Clinical history of stroke patients.

Clinical features		Total (%)
Age, *n* (%)	≤38	22 (14.8)
	>55	26 (17.2)
Gender	Male	69 (62.72)
	Female sex	41 (37.27)
Smoking history, *n* (%)	Smoking history	58 (52.72)
	No smoking history	52 (47.27)
Hypertension, *n* (%)	History of hypertension	11 (20.61)
Diabetes, *n* (%)	Diabetes history	10 (22.13)
Hyperlipidemia, *n* (%)	History of hyperlipidemia	9 (18.24)
Other diseases, *n* (%)	History of complications	6 (10.12)

**Table 2:** Comparison of upper limb FMA function results between the two groups before and after treatment (*x* ± *s*).

Group	*n*	Before treatment	After treatment
Observer	55	32.4 ± 2.5	58.6 ± 1.9
Reference group	55	30.9 ± 2.6	49.5 ± 2.1
*t* value		8.796	9.248
*P* value		0.008	0.009

**Table 3:** Comparison results of upper limb function test UEFT between the two groups (*x* ± *s*).

Group	*n*	Before nursing	After nursing
Observer	55	47.1 ± 6.5	69.8 ± 3.2
Reference group	55	40.6 ± 6.2	58.3 ± 2.5
*t* value		8.791	8.543
*P* value		0.007	0.008

**Table 4:** Comprehensive comparison of exercise ability results between the two groups.

Group	*n*	Flexibility	Fineness	Coordination
Observer	55	65.3 (71.3)	70.9 (52.4)	58.3 (51.4)
Reference group	55	50.4 (61.4)	54.2 (52.4)	49.7 (31.5)
*t* value		8.749	9.137	9.543
*P* value		0.008	0.007	0.009

## Data Availability

The data underlying the results presented in the study are available within the manuscript.
